# miR-203 Acts as a Tumor Suppressor Gene in Osteosarcoma by Regulating RAB22A

This article has been retracted.

**DOI:** 10.1371/journal.pone.0132225

**Published:** 2015-09-18

**Authors:** Dawei Yang, Guangpeng Liu, Kunzheng Wang

**Affiliations:** 1 Department of Orthopedics, The Second Affiliated Hospital of Xi’an Jiaotong University, Xi’an, 710004, Shan xi, China; 2 Department of Orthopedics, The Fourth Hospital of Harbin Medical University, Harbin 150001, Heilongjiang, China; 3 Department of Plastic and Reconstructive Surgery, Shanghai Tenth People's Hospital Tongji University School of Medicine, Shanghai, 200011, China; Sun Yat-sen University Medical School, CHINA

## Abstract

microRNAs (miRNAs), small noncoding RNAs of 19–25 nt, play an important roles in the pathological processes of tumorigenesis. The object of this study was to study the expression and function of miR-203 and to found its target gene in osteosarcoma. In our study, we found the expression level of miR-203 was significantly downregulated in osteosarcoma cell lines and tissues. In addition, overexpression of miR-203 inhibited the osteosarcoma cell proliferation and migration and inhibited Mesenchymal-to-Epithelial reversion Transition (MErT). Moreover, we identified RAB22A as a direct target of miR-203 and RAB22A overexpression blocks the roles of miR-203 in osteosarcoma cell. Furthermore, we demonstrated that RAB22A expression was upregulated in human osteosarcoma cell lines and tissues. Take together, our results demonstrated that miR-203 act as a tumor suppressor miRNA through regulating RAB22A expression and suggested its involvement in osteosarcoma progression and carcinogenesis.

## Introduction

Osteosarcoma (OS) has become the most common malignant bone tumor and occurs mainly in adolescents and young adults, which accounts for approximately 60% of malignant bone tumors in the first 2 decades of life[1–4]. It mainly present in the long bones of the body, such as the knee joint, lower femur and upper tibia in about 80% patients[5–7]. Approximately 40–50% of osteosarcoma patients will develop metastases and the main sites of metastases of OS are the lungs, pleura, and the heart[8–11]. Therefore, it is urgent to develop better prognosis, new therapeutic targets and approaches for osteosarcoma treatment.

MicroRNAs (miRNAs) are a novel series of small endogenous, non-coding, single-stranded RNAs, which negatively regulate a wide variety of genes expression mainly through direct interaction with the 3’untranslated regions (3’UTR) of their corresponding mRNA targets[12–15]. Increasing evidences have demonstrated that miRNAs play important roles in pathological and physiological processes such as cell-cycle regulation, differentiation, proliferation, apoptosis, and migration[7, 16–20]. Numerous miRNAs have been implicated in different cancers including bladder cancer, renal cell carcinoma, breast cancer, gastric cancer, playing important roles in tumorigenesis[21–26]. Therefore, miRNAs have been suggested as potential and novel targets for the diagnosis, prognosis and treatment of osteosarcoma[27, 28].

Previous studies demonstrated that miR-203 acts as a important role in various cancers[29–31]. Fox example, Liao et al[32]. reported that miR-203 expression was lower in imatinib-resistant glioblastoma (GBM) cells (U251AR, U87AR) that underwent epithelial-mesenchymal transition (EMT) than in their parental cells (U251, U87). Xu et al[33]. showed that miR-203 could be a potential prognostic marker and functions as a tumor suppressor in human renal cancer by post-transcriptionally targeting FGF2. Moreover, Lee et al[34]. demonstrated that miR-203 induces the cells apoptosis by directly targeting Yes-1 in oral cancer cells. However, the role of miR-203 in osteosarcoma is still unknown. In this study, we confirmed that the miR-203 expression is significantly decreased in osteosarcoma tissues and revealed that miR-203 could inhibit cell proliferation through directly targeting RAB22A in osteosarcoma.

## Materials and Methods

### Ethics Statement

Our experiments involving tissues were approved by the ethical board of The Second Affiliated Hospital of Xi’an Jiaotong University and complied with the Declaration of Helsinki. All of these patients gave written informed consent.

### Human tissue samples and cell lines

Osteosarcoma tissues and adjacent nontumor tissues (located 3 cm away from the tumor) were collected during surgery in our hospital. Human osteosarcoma cell lines (MG-63, SOSP-9607, SAOS-2, and U2OS) and one normal osteoblast cell line (hFOB) were purchased from the Cell Bank of Chinese Academy of Medical Sciences (Beijing, China). These cells were cultured in Dulbecco’s Modified Eagle Medium (DMEM) (Gibco).

### Oligonucleotides transfection

miR-203 mimic and negative control (scramble) were obtained from RIBOBIO (Guangzhou, China). Cells were transfected with miR-203 mimic or scramble by Lipofectamine 2000 (Invitrogen) following to the manufacturer’s instructions.

### Cell proliferation and migration assay

Cell proliferation was performed using CCKK-8 according manufacturer’sprotocol. For cell migration, a sterile white pipette tip was used to perform similar-sized wounds. Wounded cells were washed by PBS to remove cell debris and then photographed. The wound closure was measured and photographed at 0h and 48 h.

### Real-time quantitative PCR

Total RNA was extracted from tissues or cells by using TRIzol. Real-time quantitative PCR (qRT-PCR) and TaqMan microRNA assays were done to quantify the expression of mature miR-203 using SYBR Green PCR mix (Applied Biosystems) in a 7300 Real-time PCR System (Applied Biosystems). Gene expression was measured relative to U6 or GAPDH. The following primers were used: for RAB22A, (forward) 5’-TTGTAGCCATTGCAGGA-3’ and (reverse) 5’-AGGCTGTCTTCGGAGTTTGA-3’; for GAPDH, (forward) 5’-GACTCATGACCACAGTCCATGC-3’ and (reverse) 5’-AGAGGCAGGGATGATGTTCTG-3’.

### Western blot analysis

Western blot analysis was measured as described previously[35]. Total proteins were prepared from tissues or cells by using the RIPA buffer (Pierce). Protein was electrophoreses in a 10% SDS–PAGE and transferred onto membrane. Proteins were measured with anti-GAPDH and anti-RAB22A antibodies (Santa Cruz Biotechnology, Santa Cruz, CA).The signal was detected using an ECL detection system (Millipore).

### Dual luciferase reporter assay

A total of miR-203 mimic (or scramble), pGL3, RAB22A-3’UTR-WT or RAB22A-3’UTR-MUT vectors were contransfected into the MG-63 cells using Lipofectamine 2000 following to the manuscript’s instruction (Invitrogen). Relative luciferase activity was measured 48 h aftertransfection using a Dual-Luciferase Reporter kit (Promega, USA).

### Statistical analysis

Data are showed as the mean±SD. Difference between groups was analyzed using one-way ANOVA or Student’s t test. A P-value of p<0.05 was considered statistically significant.

## Result

### miR-203 was downregulated in human osteosarcoma cell lines and tissues

We examined the miR-203 levels in human osteosarcoma cell lines (MG-63, SOSP-9607, SAOS-2, and U2OS) and one normal osteoblast cell line (hFOB) using qRT-PCR and found that miR-203 expression was downregulated in human osteosarcoma cell lines compared to in hFOB(Fig 1A). Furthermore, the expression of miR-203 was downregulated in osteosarcoma tissues compared with their corresponding nontumor tissues (Fig 1B and 1C).

**Fig 1:** miR-203 was downregulated in human osteosarcoma cell lines and tissues. (A) qRT-PCR was performed to detect the miR-203 levels in human osteosarcoma cell lines (MG-63, SOSP-9607, SAOS-2, and U2OS) and one normal osteoblast cell line (hFOB). (B) qRT-PCR was performed to detect the miR-203 levels in osteosarcoma tissues and their corresponding nontumor tissues. (C) The relative expression of miR-203 was downregulated in osteosarcoma tissues compared with their corresponding nontumor tissues.

### miR-203 overexpression inhibited cell proliferation and migration

Up-regulation of miR-203 expression was discovered at 48 hours after miR-203 mimic transfection (Fig 2A). As showed in Fig 2B and 2C, miR-203 overexpression reduced cell proliferation and inhibited cell migration in the MG-63 cells.

**Fig 2:** miR-203 overexpression inhibited cell proliferation and migration. (A) qRT-PCR was performed to measure the miR-203 expression in MG-63 cells at 48 hours after miR-203 mimic transfection. (B) Overexpression of miR-203 inhibited the MG-63 cells proliferation. (C) Overexpression of miR-203 inhibited the MG-63 cells migration.

### Overexpression of miR-203 inhibited Mesenchymal-to-Epithelial reversion Transition (MErT)

We showed that overexpression of miR-203 can induce the E-cadherin mRNA expression and inhibit N-cadherin and Vimentin mRNA expression (Fig 3A). Furthermore, as determined by western blot, we also demonstrated that ectopic expression of miR-203 can enhance the protein expression of E-cadherin and inhibit the protein expression of N-cadherin and Vimentin (Fig 3B). We also found that miR-203 overexpression inhibited the mRNA expression of Twist, Snail, Slug, and Zeb1, which are the EMT transcription factors (Fig 3C).

**Fig 3:** Overexpression of miR-203 inhibited reversion of EMT. (A) Overexpression of miR-203 can induce the E-cadherin mRNA expression and inhibit N-cadherin and Vimentin mRNA expression using qRT-PCR. (B) Overexpression of miR-203 can induce the E-cadherin protein expression and inhibit N-cadherin and Vimentin protein expression using western blot. (C) The mRNA expression of Twist, Snail, Slug, and Zeb1 was analyzed by using qRT-PCR. **p<0.01 and ***p<0.001.

### miR-203 directly targets the RAB22A in osteosarcoma cells

To find the molecular mechanisms responsible for the effect of miR-203 in osteosarcoma, we used Target Scan databases to predict target genes of miR-203. We identified that RAB22A gene harbored a potential miR-203 binding site using a stringent bioinformatics approach (Fig 4A). Ectopic expression of miR-203 led to a reduction of luciferase activity when the reporter construct contained the RAB22A 3’UTR in MG-63 cells (Fig 4B). miR-203 overexpression in MG-63 cells reduced RAB22A mRNA and protein expression (Fig 4C and 4D).

**Fig 4:** miR-203 directly targets the RAB22A in osteosarcoma cells. (A) RAB22A gene harbored a potential miR-203 binding site using a stringent bioinformatics approach. (B) Ectopic expression of miR-203 led to a reduction of luciferase activity when the reporter construct contained the RAB22A 3’UTR in MG-63 cells. (C) Overexpression of miR-203 reduced RAB22A mRNA expression using qRT-PCR. (D) Overexpression of miR-203 reduced RAB22A protein expression using western blot.***p<0.001.

### RAB22A overexpression blocks the roles of miR-203

We found that RAB22A expression was upregulated in human osteosarcoma cell lines compared to in hFOB (Fig 5A). Furthermore, the expression of RAB22A was upregulated in osteosarcoma tissues compared with their corresponding nontumor tissues (Fig 5B). Western blot data confirmed that the protein expression of RAB22A was overexpressed when cells transfected with RAB22A vector (Fig 5C). We rescued the expression of RAB22A in miR-203 overexpressing MG-63 cells. CCK8 assay showed that overexpression of RAB22A increased the miR-203 overexpressing MG-63 cells proliferation (Fig 5D). Moreover, overexpression of RAB22A increased the N-cadherin and Vimentin mRNA expression and inhibited E-cadherin mRNA expression in miR-203 overexpressing MG-63 cells (Fig 5E). Furthermore, the migration abilities of miR-203 overexpressing MG-63 cells were increased after RAB22A vector transfection (Fig 5F).

**Fig 5:** RAB22A overexpression blocks the roles of miR-203. (A) qRT-PCR was performed to detect the RAB22A levels in human osteosarcoma cell lines (MG-63, SOSP-9607, SAOS-2, and U2OS) and one normal osteoblast cell line (hFOB). (B) qRT-PCR was performed to detect the RAB22A levels in osteosarcoma tissues and their corresponding nontumor tissues. (C) The protein level of RAB22A was measured using western blot. (D) CCK8 assay showed that overexpression of RAB22A increased the miR-203 overexpressing MG-63 cells proliferation. (E) The mRNA expression of E-cadherin, N-cadherin and Vimentin was measured by using qRT-PCR. (F) The migration abilities of miR-203 overexpressing MG-63 cells were increased after RAB22A vector transfection.*p<0.05 and ***p<0.001.

## Discussion

Altered patterns of miRNA expression have been well demonstrated in nearly all types of human diseases and, especially in cancers[27, 36, 37]. miRNAs are involved in tumor cell proliferation and migration by regulating numerous genes such as tumor suppressor genes and oncogenes[35, 38, 39]. In our study, we found the expression level of miR-203 was downregulated in osteosarcoma cell lines and tissues. In addition, forced overexpression of miR-203 inhibited the osteosarcoma cell proliferation and migration and inhibited MErT. Moreover, we identified RAB22A as a direct target of miR-203 and RAB22A overexpression blocks the roles of miR-203 in osteosarcoma cell. Take together, our results demonstrated that miR-203 act as a tumor suppressor miRNA and suggested its involvement in osteosarcoma progression and carcinogenesis.

Increasing data have shown that miR-203 is deregulated and functions as a tumor suppressor gene in various human cancers including cervical cancer, prostate cancer, breast cancer, colorectal cancer and glioblastoma[30, 40–43]. For example, enforced expression of miR-203 attenuated colorectal cancer cell proliferation, invasion and migration by regulating Zinc finger protein 217 (ZNF217) expression[44]. Xiang et al[45]. demonstrated that the expression of miR-203 was significantly downregulated in prostate cancer specimens and miR-203 overexpression inhibited cell proliferation, adhesion and invasion by inhibiting Rap1A expression. However, the expression and role of miR-203 in osteosarcoma is still unknown. In this study, our results showed that expression of level of miR-203 was downregulated in osteosarcoma cell lines and tissues. In addition, forced overexpression of miR-203 inhibited the osteosarcoma cell proliferation and migration and inhibited reversion of EMT. These studies may help to explain the important role of miR-203 in development and progression in osteosarcoma.

RAB22A was found as a direct target of miR-203 inosteosarcoma cells by using bioinformatics analysis, Dual luciferase reporter assay and western blot. There is a potential miR-203 binding site of RAB22A gene. Ectopic expression of miR-203 led to a reduction of luciferase activity when the reporter construct contained the RAB22A 3’UTR in MG-63 cells. Furthermore, miR-203 overexpression in MG-63 cells reduced RAB22A mRNA and protein expression. Moreover, RAB22A overexpression blocks the roles of miR-203. Furthermore, we demonstrated that RAB22A expression was upregulated in human osteosarcoma cell lines compared to in hFOB and the expression of RAB22A was upregulated in osteosarcoma tissues compared with their corresponding nontumor tissues. RAB22A belongs to a Ras superfamily of GTPases and play important roles in development of cancers[46]. Recent study has shown that RAB22A overexpression is associated with decreased overall and metastasis-free survival in the primary tumor and RAB22A knockdown impairs cancer metastasis in breast cancer[46]. Moreover, previous studies showed that miR-373 suppresses human epithelial ovarian cancer invasion and metastasis by directly targeting RAB22A gene[47]. Yang et al[48]. also reported that miR-193b as a novel tumor suppressor plays an important role in breast cancer progression by inhibiting RAB22A expression. Take together, our results showed that miR-203 may act as a tumor suppressor gene in osteosarcoma partly by regulating RAB22A expression.

In conclusion, we determined that miR-203 is downregulated in osteosarcoma cell lines and tissues, and overexpression of miR-203 inhibited osteosarcoma cell proliferation and migration via targeting RAB22A. These data demonstrated that restoration of miR-203 may be a potential therapeutic strategy for treatment of osteosarcoma.
